# Research on Cold Chain Logistics Traceability System of Fresh Agricultural Products Based on Blockchain

**DOI:** 10.1155/2022/1957957

**Published:** 2022-02-01

**Authors:** Xinghua Zhang, Yongjie Sun, Yongxin Sun

**Affiliations:** ^1^Changchun Sci-Tech University, Changchun 130600, Jilin, China; ^2^College of Life Science, Changchun Sci-Tech University, Changchun 130600, Jilin, China; ^3^College of Physics and Electronic Information, Baicheng Normal University, Baicheng 13700, Jilin, China

## Abstract

Traditional cold chain logistics has problems such as centralized data storage, low data reliability, easy data tampering, and difficulty in locating responsible persons, which leads to the inability to guarantee consumer rights. To solve these problems, a cold chain logistics traceability system is proposed for fresh agricultural products based on blockchain. Both alliance chain and private chain are used in the paper in order to ensure that the product traceability system not only has certain openness but also must contain enough privacy and security. Alliance chain is mainly used to query and share product traceability information. The private chain will be used to collect and store the product traceability information of each enterprise and then connected to the alliance chain via hash pointers. The proposed system is beneficial for reducing the burden of network transmission of alliance chain and improving the efficiency of consumer product data query. At the same time, the private chain ensures the security and privacy of enterprise product data, which not only has high data storage efficiency but also can meet the requirements of all participants for the traceability system. In the experimental part, the feasibility of this system is verified through simulation experiments, which provides a reference for the combination of blockchain technology and cold chain logistics traceability system.

## 1. Introduction

Agricultural products and cold chain logistics system from farmland to table involve production, processing, packaging, transportation, storage, sales, and other different links. Each link may have unsafe factors. In recent years, such incidents as “cadmium rice” [1], “aquatic crab,” and “smuggled frozen meat” in Guangdong [2] and “malachite green” for bass [3] and “crayfish” in Nanjing have seriously damaged the interests of consumers [4]. At the same time, the production of fresh agricultural products and cold chain logistics enterprises also suffered a heavy blow. These events further triggered a crisis of trust between consumers and fresh agricultural products enterprises [5, 6]. Traceability system has become an effective means of supply chain quality management of fresh agricultural products by reducing quality and safety risks, improving product recall efficiency, and ensuring public health [7, 8]. The research and establishment of cold chain logistics traceability system for fresh agricultural products, which can achieve effective supervision of the whole process from production to consumption, have become a hot issue of general concern.

The cold chain logistics traceability of fresh agricultural products involves agricultural supplies suppliers, farmers and other producers, processors, middlemen, and end consumers. Among them, middlemen further include logistics service providers, wholesalers, distributors, and retailers. Therefore, the cold chain logistics traceability system of fresh agricultural products is characterized by many points, long lines, wide areas, and intricate intersections [9, 10]. This makes food safety supervision and traceability particularly difficult in operation. The traditional traceability system relies on the authority to manage the central database in practice, which has the problem of data centralization. Traceability data on each supply chain node is managed by the enterprise itself and is easy to be tampered with. At the same time, the reliability of information transmission among various roles in the supply chain remains to be solved.

Blockchain technology is characterized by tamability, distribution, decentralization, traceability, and high availability. Using these characteristics of blockchain, the combination of blockchain technology and cold chain logistics traceability of fresh agricultural products provides the possibility of solving the problems existing in the current traditional agricultural products traceability system. In recent years, domestic and foreign scholars [11–14] have carried out exploration and research in the field of agricultural product traceability. The existing methods are mostly based on the existing common blockchain systems such as Bitcoin, Ethereum, and Hyperledger Fabric system for application development. They have some bottleneck problems in data storage, such as low query efficiency, high data storage pressure, and poor data security. In practical applications, the following problems may occur when blockchain is used as a data management platform for traceability applications. As the quantity of nodes and data increases, the underlying storage system is frequently accessed by users. This puts forward high requirements on the function and performance of the data storage system.

Therefore, this paper proposed a cold chain logistics traceability system of fresh agricultural products based on blockchain, which is from the perspective of improving the efficient information storage and fast query efficiency of the cold chain logistics traceability system of fresh agricultural products. In order to ensure the high reliability of blockchain operation environment, the traceability system adopts the dual chain structure design of alliance chain and private chain. In the experiment, the feasibility of the system is verified by simulation experiment.

## 2. Related Work

### 2.1. Traceability to the Safety of Cold Chain Logistics

Cold chain logistics generally refers to system engineering to ensure product quality and reduce product loss, keeping refrigerated and frozen products in a specified low temperature environment all the time. Production, storage, transportation, distribution, sales, and consumption before the purchase of each link are included among them. Studies have found that every 6° increase in temperature will double the growth rate of bacteria in food and shorten the shelf life by half [15]. When ambient temperatures rise at any point, bacteria multiply more quickly. This is the impact of temperature change on food safety that most people are not aware of.

The essence of traceability is to turn the physical circulation of industrial chain into information flow. The production and circulation information of products can be obtained according to the tracking and query of information flow [16]. Agricultural product safety traceability refers to the ability to track the flow of products when there are safety problems in agricultural products, then recall the problematic food, cut off the source, and eliminate the harm. Therefore, each link needs to record the corresponding information from the production, circulation, and final consumption of agricultural products. For consumers, traceable agricultural products provide transparent product information. This enables consumers to fully enjoy the right to know when buying and to make the right purchase choice. It has always been regarded as the most complicated and difficult part of food traceability because of the wide circulation range, long chain, and many links of agricultural products.

The accurate and real-time whole process record provided by cold chain logistics provides conditions to trace agricultural product information accurately and effectively. The working principle of cold chain logistics relies on modern information technology with the help of advanced management methods and organization. Typically, a combination of RFID (Radio Frequency Identification), GPS (Global Positioning System), GIS (Geographic Information System), mobile communications, and temperature sensing technology is used [17]. Then, the record of temperature and humidity change is uploaded to the management platform for real-time management of product quality. This intelligent, information-based cold chain logistics process provides technical support for agricultural products traceability. However, in order to complete the traceability management of agricultural products, it is necessary to establish the necessary basic information base for its core information such as planting, storage, processing and distribution, sales, and consumer attention. Through the information management platform, the discovered problems can be queried, and the generated problems can be held accountable.

### 2.2. Basic Introduction to Blockchain

#### 2.2.1. Blockchain

Blockchain is a chain structure of blocks of data arranged in chronological order through cryptography algorithms. It can realize decentralized, tamper-proof, traceable, and multiparty jointly maintained distributed database [18]. Each party must agree to update the data according to the pre-agreed rules and implement information sharing and monitoring among the parties. Blockchain integrates P2P network, cryptography [19], smart contract [20], consensus mechanism [21], timestamp [22], blockchain structure, and other technologies. It can realize self-verification and management of data without relying on third parties.

#### 2.2.2. Block Structure

Blockchain is an ordered chain of data block structure with block as unit, and each block is composed of block head and block body [23]. As shown in Figure 1, each block header contains the hash value of the previous block header. The original block is connected to the current block and forms a chained data storage structure. The properties of the Merkle tree structure and the connection between timestamps and blocks are utilized to ensure that each block is connected chronologically and the data is not susceptible to tampering [24]. Even if it is tampered with, it can be quickly located, which ensures the reliability and credibility of the traceability system data [25].

#### 2.2.3. Hash Algorithm

The hash algorithm can map data of any length to a short-fixed length binary value through hash function [26, 27]. It is an irreversible mapping from plaintext to ciphertext; that is, the same input always yields the same output. Using the characteristics of hash function, it can not only verify whether trace data is tampered with, but also ensure the security of data. In practical applications, MD5 [28] algorithm is usually adopted, which generates a 32-bit hexadecimal sequence value for the input of arbitrary length string.

#### 2.2.4. Blockchain Classification

According to the degree of regional decentralization, blockchain is mainly divided into public chain, alliance chain, and private chain [29]. In the traceability system, the responsible subjects of the agricultural supply chain belong to the cooperative relationship, but at the same time, they cannot be completely trusted. There is already association, horizontal interconnection and cooperation, or vertical transaction relationship. Therefore, alliance chain is usually used as the technical framework for agricultural product traceability system research [30].

## 3. The Proposed Model in This Paper

### 3.1. Cold Chain Logistics Process Analysis of Fresh Agricultural Products

In order to design the traceability system of fresh agricultural products, the management mode of its generation to sales will be analyzed first, and then the traceability management method will be designed according to the characteristics of each link. The main body of “base + supermarket” agricultural cold chain logistics is clear, and the key points of traceability information flow are easy to define compared with other complex and diverse circulation forms of agricultural products. The specific process is as follows.

#### 3.1.1. Planting and Harvesting

When agricultural products are still in the “field,” their growth process will suffer from the soil pesticide residues, heavy metals, and other irreversible harm. Improper fertilization can also cause quality problems in agricultural products. Therefore, all production plots and greenhouses need to be numbered uniformly. The turnover box of picking agricultural products should also be managed by numbering, and strict and accurate records should be made. The harvest time of agricultural products is short, and the process has little impact on the quality of agricultural products. In this stage, process records and quality testing reports are mainly carried out.

#### 3.1.2. Storage and Processing

Harvested agricultural products that are not immediately listed need to be stored or circulated for processing. This link should strengthen production monitoring. The agricultural products cold storage requirements and the absolute safety of processing are ensured, depending on the temperature sensing technology. In this link, records of storage temperature, humidity, processing, and storage time should be made.

#### 3.1.3. Transportation and Distribution

Transport vehicles for agricultural products shall comply with health requirements and be equipped with a continuous output of temperature records that cannot be artificially altered. The docking of agricultural product information should be carried out before transportation and distribution. In the process of distribution and transportation, GPS and GIS should be relied on to track and monitor the situation of agricultural products and refrigerated vehicles. This is to prevent damage to agricultural products caused by improper handling or microbial damage. In this link, records of transportation temperature, humidity, geographical location, and transportation time should be made. The logistics information recording process is shown in Figure 2.

#### 3.1.4. Supermarket Sales

The sales of agricultural products still need refrigeration preservation technology to ensure the quality of agricultural products, which usually should be displayed and sold in accordance with the storage temperature and humidity of agricultural products. In this link, the refrigeration temperature, humidity, purchase and sale time, and other information should be well recorded.

The record of the above key points provides the prerequisite for the establishment of agricultural products traceability system. First, base operators generate retrospective two-dimensional code for the harvested agricultural products according to the production number and paste it on the packaging of agricultural products. The additional information is mainly the production experience of agricultural products, for example, the planting date; the fertilization date; the fertilization duration; and the use of pesticides, growth promoters, and other related auxiliary products. Record the names; sources; users; and pickers of pesticides, fertilizers, and regulators used. Upload production file information to the platform through information technology. In the subsequent cold chain logistics, the storage file, transportation file, and distribution file of each link should be recorded. Then, the cold chain logistics operator will upload them to the platform in real time. Finally, consumers who buy products at a supermarket scan a QR code on the package. Users can query the detailed information and quality test report of agricultural products from planting, production, transportation, storage, and sales through the platform. At the same time, the upstream subject can also track the information of agricultural products in each link of circulation through the platform. The traceability system of “base + supermarket” agricultural cold chain logistics integrates the records of planting, collection, and key points of cold chain logistics into the database information of the traceability system. Through the operation of the traceability service management platform, the main body of the agricultural supply chain can share information and achieve convenient and accurate traceability of agricultural products.

### 3.2. Data Structure of Private Chain and Alliance Chain

#### 3.2.1. Participant Setting of the Anticounterfeiting Traceability System

The function and nature of product traceability determine that it has many participants, mainly including various manufacturers, relevant national departments, and consumers. Product traceability system must contain sufficient privacy and security while requiring certain openness. This paper proposes an anticounterfeiting traceability system using both alliance chain and private chain. The alliance chain is mainly used to query and share product traceability information. The private chain will be used to collect and store the product traceability information of each enterprise and then connected to the alliance chain through the hash pointer. This design method is beneficial for reducing the burden of network transmission of alliance chain and improving the efficiency of consumer product data query. The private chain ensures the security and privacy of enterprise product data. It not only has high data storage efficiency, but also can meet the requirements of all participants for the traceability system. The production department, transportation and storage department, sales department, information technology department, and national supervision department of each enterprise jointly maintain the private chain and add product traceability information and audit information of the supervision department to the private chain. Among them, the state supervision department, as the organizer of the private chain, will participate in the audit and authorization of enterprises. The information technology department is responsible for collecting information packaging blocks as the holder of billing rights for the private chain. Other departments in each enterprise and national law enforcement departments jointly maintain the alliance chain and provide external tracing information query function.

#### 3.2.2. Product Traceability Information Structure

Blockchain does not prevent the initial data fraud; that is, it does not prevent companies from falsifying product raw materials, warehousing, and other information. Thus, companies will use IoT (Internet of Things) technology to monitor production, processing, and warehousing in real time and establish a set of intelligent production lines and storage lines to ensure the authenticity of the source data reliability.

As shown in Table 1, for a certain product, the production information *P* generated by the production department of the enterprise includes but is not limited to product ID, product name, raw material information (recorded by sensors and transmitted to the production department), signature *S*_*x*_ of the person in charge, and hash value *H*(*P*) of the production information.

As shown in Table 2, for a certain product, the transportation and storage information *T* generated by the transportation and storage department of the enterprise includes but is not limited to transportation time, transportation mode, storage information (transmitted through temperature sensors, etc.), signature *S*_*y*_ of the person in charge, and hash value *H*(*T*) of the transportation and storage information.

As shown in Table 3, for a certain product, sales information *S* generated by the sales department of the enterprise includes but is not limited to sales time, sales quantity, sales method, signature *S*_*z*_ of the person in charge, and hash value *H*(*S*) of sales information *S*.

In order to prevent enterprises from tampering with their product traceability information, the above three types of traceability information should also be submitted to the national regulatory authorities for audit, and the audit information *C* can be obtained. Using the input sensitive property of hash function, check whether trace information is tampered with. In case of alteration, responsibility can be quickly confirmed according to the signature of the person in charge in each process to prevent the circulation of illegal products. If there is no alteration, it will be handled by the enterprise information technology department.

After the examination and verification by the national supervision department, the information technology department of the enterprise shall collect production information *P*, transportation and storage information *T*, sales information *S*, and audit information *C*, and then *S*_*i*_ is signed by the head of the information technology department. A transaction in a private chain block, the structure of which is shown in Table 4 is constituted.

After the above procedure is performed, a secure and reliable private chain of product traceability information will be generated. In order to prevent the leakage of enterprise privacy data, enterprises can only query the information of their own products on the private chain. Due to the large amount of data transmitted in the private chain, it is not suitable for transmission in the alliance chain that provides the query function. Therefore, it is not necessary to store complete product traceability information in the alliance chain block body, but to store the block header hash value of each block in the private chain. This can improve the efficiency of data transmission in the alliance chain. At the same time, according to the characteristics of Merkle tree and hash function, product traceability information items will correspond one by one, and there is no confusion of traceability information. The header of the block in the alliance chain consists of the current block hash, the hash of the previous block header, the timestamp, the Merkle root, and the associated responsible signature. The block body contains the hash value of each block header in the private chain.  Figure 3 shows the data structure of the private and alliance chains.

### 3.3. The Proposed Cold Chain Logistics Traceability System

#### 3.3.1. Storage Mechanism Design

There are many participating nodes in the blockchain-based agricultural supply chain, and the data collection volume of nodes in each link is large. If all the nodes are uploaded to the blockchain network at one time, in addition to the slow upload speed, the operation cost will be greatly increased, and the hardware requirements for nodes in each link will be high. Therefore, the dual-storage mechanism will be adopted in this paper; that is, the collected data information of nodes in each link will be stored together in the blockchain network and the relational database. However, the summary of information generated by SHA-3 (Secure Hash Algorithm 3) is stored in the blockchain network, while the complete information is stored in the database. This not only improves the operational efficiency of blockchain, but also solves the scalability problem faced by blockchain.

#### 3.3.2. Design of the Traceability System of Fresh Agricultural Products

After the above process analysis and storage mechanism design of agricultural supply chain, the structure diagram of agricultural product traceability scheme is designed, as shown in Figure 4.

The data stored in the traceability solution is stored by the blockchain system and the database. Introducing the relational database can solve the scalability problem of the blockchain system. Only a summary of the data is stored in a blockchain system, and the complete data is stored in a database. The database is maintained by the Administration for Industry and Commerce, while the blockchain system is jointly maintained by production enterprises, transportation enterprises, warehouse storage enterprises, sales enterprises, Food and Drug Administration, and Industry and Commerce Administration. The original intention of this system is to provide traceability inquiry services for consumers and provide more convenient and efficient supervision services for the regulatory authorities, so it also includes external users such as the regulatory authorities and consumers.

The information input process of the production enterprise, transportation enterprise, warehouse storage enterprise, and sales enterprise is the same. Taking the production enterprise as an example, the production enterprise packages the collected data and inputs it into the node and database at the same time. The production enterprise node generates a summary of the input data using SHA-3 and sends it to the blockchain. After reaching a consensus, the participating nodes write a summary of the information into the block. At this point, the block returns a hash value to be stored in the database, which can be used for data indexing. The Administration for Industry and Commerce and the Food and Drug Administration supervise the behavior of the above nodes.

Consumers purchasing food can use the code on the package in the database for traceability inquiry. If you have doubts about the queried information, you can query and compare the summary of the information in the blockchain to determine whether the data has been changed. If the information summaries are consistent, the data is true and unchanged. When it is found that the query data has been changed, consumers can complain to the Administration for Industry and Commerce. The complaint information will be stored in the database and blockchain system in the same way as evidence.

Due to the large amount of data collected in each link of the agricultural supply chain, information may be omitted or incorrectly recorded due to manual error or other external interference during information input. In addition, once the information is entered into the blockchain system, the data cannot be changed, so the Food and Drug Administration is introduced into this scheme. If any node in the agricultural supply chain finds any error in the input information, it can send an information correction request to the Food and Drug Administration. After being verified by the Food and Drug Administration, the corrected information can be uploaded to the blockchain system by the FDA node. These methods can eliminate the huge loss of information input errors caused by human operation errors.

The design of agricultural product traceability scheme based on blockchain ensures that data cannot be tampered with and the centralized structure is removed. The traceability of information flow has realized the function of quick search and accurate positioning. According to the actual needs of targeted introduction of Food and Drug Administration and Industry and Commerce Administration. The Food and Drug Administration can not only deal with information entry errors at all stages of the supply chain, but also provide data correction needs. It can also recall problematic food that may cause damage to human health. The Administration for Industry and Commerce is responsible for the timely acceptance of consumer complaints. Information about complaints that may damage consumers' health will be shared with the Food and Drug Administration in a timely manner, carrying out food recall work in a timely manner.

#### 3.3.3. Traceability Architecture Based on Blockchain

Figure 5 shows the traceability system hierarchy based on blockchain. The architecture is mainly divided into six layers from bottom to top, namely, operation layer, data acquisition layer, data layer, consensus and network layer, presentation layer, and user layer. The bottom layer is the operation layer, which refers to the production enterprises, transportation enterprises, warehouse storage enterprises, and sales enterprises that need to collect data. It is the source of the entire traceability data. Data acquisition layer refers to the use of radio frequency devices, information acquisition terminals, and application sensors to collect and transmit data at the operation layer and can improve the overall efficiency of agricultural supply chain. The data layer transfers data from the data acquisition layer to the data storage layer. It adopts the dual blockchain mechanism of alliance chain and private chain. Only a summary of the processed information is stored in a blockchain network, while the complete data and the hash values returned after the summarization are stored in a relational database. Consensus and network layer refers to key technologies of blockchain including P2P network, authentication mechanism, propagation mechanism, and PoW and PoS consensus mechanism. Presentation layer refers to the use of B/S architecture and JSP (Java Server Pages) technology to display data according to user needs. The top layer is the user layer, including production enterprises, transportation enterprises, warehouse storage enterprises, sales enterprises, regulatory departments, and consumers. Production enterprises, transportation enterprises, warehouse storage enterprises, and sales enterprises are responsible for information entry. Regulatory authorities and consumers can query product information in the system according to their needs.

## 4. Experiment

### 4.1. Experimental Environment

In this simulation experiment, three PCs are mainly used to achieve traceability by building simulation private chain, alliance chain, and traceability platform. The experimental environment is shown in Table 5. The test is conducted in virtual machine simulation test, and its environment is based on CentOS 8.0. The operating memory is 8 GB, the hard disk is 500 GB, and the bandwidth is 200 Mb/s. The Fabric network contains four Peer nodes and one Orderer node. The default LevelDB database in the Fabric has a single query form. CouchDB meets real world needs and supports rich queries. Composite keys are modeled to support equivalent queries for multiple parameters. Therefore, this paper chooses CouchDB as the test database. Node SDK was used to develop test programs, and REST interface was used to call resources.

### 4.2. Analysis of Data Generation Efficiency

In the experiment, a simple private chain system was built on PC1 to store detailed product traceability data, in which raw material information and storage information were roughly represented as product origin and raw material storage place. The traceability data of 20 kinds of products are simulated in the experiment, and the traceability function is realized by connecting them together according to previous_hash. At the same time, any modification of the data will destroy the chain structure and ensure that the data cannot be modified by changing.

Then, a simple alliance chain system is built on PC2 to store the hash value of the block header of the private chain.

Finally, a small product information traceability platform is built on PC3, and its data sources are from private chain and alliance chain. For the query of the traceability data of a product, the system will automatically take its hash value after the user enters the commodity name and then turn it over to the relevant block of the private chain for search after the processing of the alliance chain. The data will be returned to the platform matching request first and then to the user data. If the traceability information is not found, the user can submit feedback.

In terms of system performance, the running time of the anticounterfeiting traceability system proposed in this paper is mainly spent on the collection, transmission, and audit of traceability data. In the process of generating traceability data, the sensor can transmit accurate data in real time and consume less time. In addition, the information generated by each department depends mainly on network factors. As shown in Figure 6, under common network conditions, the system built in this paper was tested 20 times, in which the generation time of private chain transaction data ranged from 524 to 890 ms, with an average of 632 ms. The generation time of alliance chain transaction data ranged from 513 to 73 ms, with an average of 617 ms.

### 4.3. Query Efficiency Analysis

Based on realizing the design of the above traceability system, it is necessary to show the information of the growth and circulation of agricultural products to consumers. Therefore, it is necessary to quickly trace the information of agricultural products batch. According to the different ways of storing blockchain traceability data, there are two commonly used query methods as follows:

1. The first method is the key traversal query, namely, key method. Data information items about the growth, processing, logistics, and sales of agricultural products will be written into the blockchain one by one. The ID of the traceability information is used as the key value, and the traceability information is stored in the blockchain as the value. The key is used as the index to traverse the previous block from the latest block to obtain the matching value during querying the traceability information. In addition to the fresh agricultural product traceability business, there are multiple traceability information uploading records of agricultural product batches. Batch information is usually obtained during query, requiring multiple traversals of the block by key. The number of iterations is related to the number of agricultural products batch traceability records.
2. The second method is to query information by the field of batch number, namely, batch method. Specifically, the growth, processing, logistics, and sales of agricultural products are written into the blockchain. The ID of the traceability information is used as the key value, and the traceability information is stored in the blockchain as the value. The query uses CouchDB's rich query to traverse from the latest block to the previous block by the batch number field in value. To obtain all the traceability information of a batch of agricultural products, you only need to traverse all blocks once to get all the traceability information of a batch of agricultural products.

This paper tests and compares the above two query methods. During the experiment, the same query operation is executed under the same circumstances, and the query time will fluctuate in a certain range. To ensure the objectivity of the data, each set of data is executed 10 times, and its average is calculated as the final value. The above methods were used to test the experiment, and the correlation analysis of the test results was carried out. The correlation coefficient can be calculated by

(1) $$\begin{array}{c} R_{\left(X,Y\right)}=\frac{\text{Cov}\left(X,Y\right)}{\sqrt{D\left(X\right)}\sqrt{D\left(Y\right)}}, \end{array}$$

where Cov(*X*, *Y*) is the covariance of *X* and *Y*. *D*(*X*) and *D*(*Y*) are the variances of *X* and *Y*, respectively.

The comparison diagram of the relationship between the query time and the number of trace records under the specific total amount of trace records for these two query methods is shown in Figure 7. Figures 7(a)-7(c) show the comparison of query time in two different ways when the total number of retrospective records is 1x10^4^, 5x10^4^, and 9x10^4^, respectively. The abscissa is the number of batch traceability records, which is 1, 200, 400, 600, 800, and 1000. The ordinate indicates the time it takes to query information. *R* represents correlation coefficient. Among them, the query time of key method is positively correlated with the number of batch traceability records. Correlation coefficients *R* were all >0.89. However, the correlation coefficients of time and trace records by batch method were all <0.5, showing a weak correlation.

Based on the above correlation analysis, the query efficiency improvement rate of the two methods is further analyzed, and its calculation equation is

(2) $$\begin{array}{c} n_{\left(\text{A},\text{B}\right)}=\frac{t_{\text{B}}-t_{\text{A}}}{t_{\text{B}}}\times 100\text{\%,} \end{array}$$

where *n*_(A, B)_ represents the efficiency improvement rate of A over B. *t*_B_ and *t*_A_ represent the time required by A and B, respectively.

As can be seen from Table 6, when querying a single traceability record, the query efficiency of batch query method fluctuates compared with that of key method. This is because the time required by a single query is small and the data fluctuation interval is large, resulting in a large difference in query time. When the number of batch traceability records is more than 200, the query efficiency of batch query method is basically stable at 60.77%–72.42% compared with key method. In practice, agricultural product batches are recorded in the range of 200–400, while the total number of traceability records in the blockchain system increases with each node and time. When the number of batch traceability records is 200, and the total number of traceability records is 1 × 10⁴, 3 × 10⁴, 5 × 10⁴, 7 × 10⁴, 9 × 10⁴, and 11 × 10⁴, the query efficiency of batch method is improved by 70.77%, 71.43%, 69.53%, 69.58%, 69.2%, and 67.73%, respectively, compared with key method. When the number of batch traceability records is 400 and the total number of traceability records is 1 × 10⁴, 3 × 10⁴, 5 × 10⁴, 7 × 10⁴, 9 × 10⁴, and 11 × 10⁴, the query efficiency of batch method is improved by 70.35%, 73.33%, 70.91%, 69.82%, 69.16%, and 71.57%, respectively, compared with key method. From the perspective of the number of batch traceability records, the query efficiency of the content query method increases with the increase of the total number of traceability records.

### 4.4. System Security Analysis

The anticounterfeiting traceability system based on double blockchain and Internet of Things technology proposed in this paper has strong security, which is mainly reflected in the following aspects:

1. Any modification of product traceability data will inevitably break the blockchain chain structure based on the security of blockchain itself, such as decentralization, immutability, and high fault tolerance. This increases the cost and difficulty of data modification and ensures the authenticity and reliability of traceability data. At the same time, it can also urge enterprises not to fabricate information in the process of product production to a certain extent.
2. Use the Internet of Things technology to generate real and objective product data and transfer it to the product data of relevant departments to block the possibility of data source fraud. This measure improves the security and reliability of product traceability data.
3. The double-chain structure of alliance chain and private chain can ensure the high reliability of blockchain operation environment. Alliance chains and private chains are built, deployed, and run based on a trusted partnership. All participants are vetted before joining the blockchain network, which greatly reduces the possibility of malicious nodes in the system. This can also prevent internal attacks, further improving the security of the system.

## 5. Conclusion

On the premise that more and more people pay attention to product safety, many problems of traditional product traceability system, such as centralized storage, low reliability of data, easy data tampering, and difficulty in locating the responsible person, are analyzed in this paper. Besides, the related work of other scholars in the field of product traceability is sorted out, and the characteristics of information traceability and non-tampering of blockchain technology are expounded. In order to solve the security and privacy problems in the cold chain logistics traceability system of fresh agricultural products, a traceability system based on blockchain is proposed in the paper. Specific work includes the following: (1) The whole process of cold chain logistics of fresh agricultural products is systematically analyzed. (2) The data structure of private chain and alliance chain is analyzed. (3) Logistics traceability system based on private chain and alliance chain is designed. The alliance chain is mainly used to query and share product traceability information. The private chain will be used to collect and store the product traceability information of each enterprise and then connected to the federation chain via hash pointers. The feasibility of this system is verified by simulation experiments, which provides reference for the combination of blockchain technology and cold chain logistics traceability system. At present, the product anticounterfeiting traceability system using blockchain technology is still in the initial stage of exploration, and its applicable product types need further analysis. There are also some security issues with its integration with the Internet of Things. The next step will continue to refine the details of the combination of the two and improve the product traceability system.

## Figures and Tables

**Figure 1:** Structure diagram of block data.

**Figure 2:** Logistics information recording process.

**Figure 3:** Data structure of private chain and alliance chain.

**Figure 4:** Structure of the proposed traceability system.

**Figure 5:** Hierarchy diagram of the proposed traceability system.

**Figure 6:** Time of data generation.

**Figure 7:** Time comparison between the two query methods.

**Table 1:** Production information.

Product ID	Product name	Raw material information	*S*_*x*_	*H*(*P*)

**Table 2:** Transportation and storage information.

Transportation time	The mode of transportation	Storage information	*S*_*y*_	*H*(*T*)

**Table 3:** Sales information.

Sales time	The sales amount	Sales way	*S*_*z*_	*H*(*S*)

**Table 4:** Private chain transaction structure.

Production information *P*	Transport warehouse information *T*	Sales information *S*	Audit information *C*	*S*_*i*_

**Table 5:** Description of experimental environment.

Name	CPU/memory	Operating system	Main function
PC1	i7-9700/8 GB	CentOS 8.0	Deploying private chains
PC2	i7-9700/8 GB	CentOS 8.0	Deploying alliance chain
PC3	i7-9700/8 GB	CentOS 8.0	Building traceability platform

**Table 6:** Percentage of efficiency improvement.

Total traceability record	Number of batch total traceability records (batch method is compared with key method)					
	1 × 10⁴	3 × 10⁴	5 × 10⁴	7 × 10⁴	9 × 10⁴	11 × 10⁴
1	34.07	7.1	11.96	8.86	21.78	-22.37
200	70.77	71.43	69.53	69.58	69.2	67.73
400	70.35	73.33	70.91	69.82	69.16	71.57
600	69.98	70.43	70.3	64.87	69.85	70.34
800	70.85	71.08	70.78	68.96	72.42	71.38
1000	60.77	68.74	64.21	61.92	60.23	65.85

## Data Availability

The labeled dataset used to support the findings of this study is available from the corresponding author upon request.

## References

[1] Wen Y., Li W., Yang Z., Guo C., Ji J. (2020). Evaluation of various approaches to predict cadmium bioavailability to rice grown in soils with high geochemical background in the karst region, Southwestern China[J]. *Environmental Pollution*.

[2] Vergne T., Chen-Fu C., Li S. (2017). Pig empire under infectious threat: risk of African swine fever introduction into the People’s Republic of China[J]. *The Veterinary Record*.

[3] Li L., Peng A., Lin Z., Zhong H. P., Chen X. M. (2017). Biomimetic ELISA detection of malachite green based on molecularly imprinted polymer film[J]. *Food Chemistry*.

[4] Guo B., Xie G., Li X. (2019). Outbreak of Haff disease caused by consumption of crayfish (*Procambarus clarkii*) in Nanjing, China[J]. *Clinical Toxicology*.

[5] Jin S., Zhang Y., Xu Y. (2017). Amount of information and the willingness of consumers to pay for food traceability in China[J]. *Food Control*.

[6] Qian J., Ruiz-Garcia L., Fan B. (2020). Food traceability system from governmental, corporate, and consumer perspectives in the European Union and China: a comparative review[J]. *Trends in Food Science & Technology*.

[7] Tian F. A supply chain traceability system for food safety based on HACCP, blockchain & Internet of things.

[8] Cruz Introini S., Boza A., Alemany Díaz M. D. M. (2018). Traceability in the food supply chain: review of the literature from a technological perspective[J]. *Dirección y Organización*.

[9] Liao Y., Xu K. (2019). Traceability system of agricultural product based on block-chain and application in tea quality safety management[C]//Journal of Physics: conference Series. *IOP Publishing*.

[10] Wongpatikaseree K., Kanka P., Ratikan A. Developing smart farm and traceability system for agricultural products using IoT technology.

[11] Hua J., Wang X., Kang M., Wang H., Wang F. Y. Blockchain based provenance for agricultural products: a distributed platform with duplicated and shared bookkeeping.

[12] Salah K., Nizamuddin N., Jayaraman R., Omar M. (2019). Blockchain-based soybean traceability in agricultural supply chain[J]. *IEEE Access*.

[13] Prashar D., Jha N., Jha S., Lee Y., Joshi G. P. (2020). Blockchain-based traceability and visibility for agricultural products: a decentralized way of ensuring food safety in India[J]. *Sustainability*.

[14] Li J., Wang X. Research on the application of blockchain in the traceability system of agricultural products.

[15] Longo F., Nicoletti L., Padovano A. (2020). Estimating the impact of blockchain adoption in the food processing industry and supply chain[J]. *International Journal of Food Engineering*.

[16] Dasaklis T. K., Casino F., Patsakis C. Defining granularity levels for supply chain traceability based on IoT and blockchain.

[17] Chen C. L., Lim Z. Y., Liao H. C., Deng Y. Y., Chen P. (2021). A traceable and verifiable tobacco products logistics system with GPS and RFID technologies[J]. *Applied Sciences*.

[18] Shao Q. F., Jin C. Q., Zhang Z., Qian W. N. (2018). Blockchain, architecture and research progress[J]. *Chinese Journal of Computers*.

[19] Fernando E., Agustin D., Irsan M., Murad D. F., Rohayani H., Sujana D. Performance comparison of symmetries encryption algorithm AES and DES with raspberry pi.

[20] Mohanta B. K., Panda S. S., Jena D. An overview of smart contract and use cases in blockchain technology.

[21] Alfandi O., Otoum S., Jararweh Y. Blockchain solution for iot-based critical infrastructures: byzantine fault tolerance.

[22] Zhang Y., Xu C., Cheng N., Yang H., Shen X. (2019). Chronos+: an accurate blockchain-based time-stamping scheme for cloud storage[J]. *IEEE Transactions on Services Computing*.

[23] Lu Y. (2019). The blockchain: state-of-the-art and research challenges[J]. *Journal of Industrial Information Integration*.

[24] Zhu H., Guo Y., Zhang L. (2021). An improved convolution Merkle tree-based blockchain electronic medical record secure storage scheme[J]. *Journal of Information Security and Applications*.

[25] He P., Yu G., Zhang Y. F. (2017). Survey on blockchain technology and its application prospects[J]. *Computer Science*.

[26] Ajao L. A., Agajo J., Adedokun E. A., Karngong L. (2019). Crypto hash algorithm-based blockchain technology for managing decentralized ledger database in oil and gas industry. *D-J Series*.

[27] Seok B., Park J., Park J. H. (2019). A lightweight hash-based blockchain architecture for industrial IoT[J]. *Applied Sciences*.

[28] Yaji S., Bangera K., Neelima B. Privacy preserving in blockchain based on partial homomorphic encryption system for AI applications.

[29] Xia X., Lin X., Dong W., He Z. (2019). Design of traceability system for medical devices based on blockchain. *Journal of Physics: Conference Series*.

[30] Xie W., Zheng X., Lu X., Lin X., Fan X. Agricultural product traceability system based on blockchain technology.

